# Ethnogynaecological Knowledge of Traditional Medicinal Plants Used by the Indigenous Communities of North Waziristan, Pakistan

**DOI:** 10.1155/2022/6528264

**Published:** 2022-08-04

**Authors:** Sabith Rehman, Zafar Iqbal, Rahmatullah Qureshi, Inayat Ur Rahman, Muazzam Ali Khan, Mohamed M. A. Elshaer, Dunia A. Al Farraj, Mohamed S. Elshikh, Muhammad Younas, Shazia Sakhi, Ghazala Nawaz, Niaz Ali, Fazal Rahim, Hamid Ali, Imran Khan, Siddiq Ur Rahman, Noha M. Abu Bakr Elsaid

**Affiliations:** ^1^Department of Botany, Hazara University, Mansehra 21300, Khyber Pakhtunkhwa, Pakistan; ^2^Department of Botany, PMAS-Arid Agriculture University, Rawalpindi, Pakistan; ^3^William L. Brown Center, Missouri Botanical Garden, 4344 Shaw Blvd, St. Louis, MO 63110, USA; ^4^Department of Botany, Khushal Khan Khattak University, Karak, KP, Pakistan; ^5^Department of Botany, Bacha Khan University, Charsada, KP, Pakistan; ^6^Department of Clinical Pharmacology, Faculty of Medicine, Ain Shams University, Cairo 11566, Egypt; ^7^Department of Clinical Pharmacology, Faculty of Medicine, King Salman International University, South Sinai 46511, El Tor, Egypt; ^8^Department of Botany and Microbiology, College of Science, King Saud University, P. No. 2455, Riyadh 11451, Saudi Arabia; ^9^Center of Plant Sciences and Biodiversity, University of Swat, Swat, KP, Pakistan; ^10^Department of Botany, Kohat University of Science & Technology, Kohat, KP, Pakistan; ^11^Department of Biotechnology & Genetic Engineering, Hazara University, Mansehra, KP, Pakistan; ^12^College of Bioscience and Biotechnology, Yangzhou University, Yangzhou 225009, China; ^13^Department of Computer Science & Bioinformatics, Khushal Khan Khattak University, Karak, KP, Pakistan; ^14^Department of Public Health, Community, Environmental and Occupational Medicine, Faculty of Medicine, Suez Canal University, Ismailia 41511, Egypt; ^15^Department of Basic Medical Sciences, Faculty of Medicine, King Salman International University, South Sinai 46511, El Tor, Egypt

## Abstract

**Background:**

Since the beginning of civilization, medicinal plants have been used in human healthcare systems. Studies have been conducted worldwide to evaluate their efficacy, and some of the results have triggered the development of plant-based medications. Rural women in Pakistan frequently experience gynaecological disorders due to malnutrition and heavy physical work during pregnancy. Due to the low economic status, the remoteness of the area, and the lack of modern health services, herbal therapy for gynaecological disorders is common among the indigenous tribes of the study area.

**Methods:**

Field surveys were carried out from April 2018 to October 2020 to collect data regarding medicinal plants used for different gynaecological disorders. A semistructured questionnaire was used to collect ethnogynaecological data.

**Results:**

In total, 67 medicinal plant species belonging to 38 families are being used to treat 26 different gynaecological problems. The herbaceous growth form and the Lamiaceae family were recorded with the maximum number of plant species (42 species and 7 species, respectively). Leaves are the most highly utilized plant part, with 16 species. In the case preparation method, decoction was the dominant method (25 species, 36.76%). The informants reported the maximum number of species for the treatment of irregular menstrual flow as 11 species (15.28%). The highest relative frequency of citation (RFC) value was obtained for *Acacia modesta* (0.37), and the use value (UV) for *Tecomella undulata* (0.85). The highest informants' consensus factor (ICF) value (1.0) was obtained for emmenagogue and tonic each after delivery. The highest consensus index (CI%) value was calculated for *Acacia modesta* (36.92%). The Lamiaceae had the highest family importance value (FIV) (98.46%).

**Conclusion:**

This is the first ever quantitative study focusing mainly on ethnogynaecological study conducted in the tribal areas of North Waziristan which highlights the importance of traditional herbal remedies for their basic medical requirements. The results of this study would serve as a baseline for advanced phytochemical and pharmacological screening, as well as conservationists for further studies.

## 1. Introduction

Ethnogynaecology is a new branch of ethnobotany, which mainly deals with the use of therapeutic plants for curing gynaecological disorders such as menses problems, abortion, lactation, infertility, gonorrhea, leucorrhoea, and delivery disorders [1, 2]. It has been documented that sexual and other women's basic healthcare problems are reported to account for 18% of the total worldwide diseases [3]. Medicinal plants used to treat gynaecological disorders such as menstrual pain, abortion, leucorrhoea, pregnancy, infertility, lactation, and delivery problems have been documented in some areas of this region's ethnic groups [4]. The tribal communities have been preparing medication from the available medicinal plant species, which are widely used to cure common women's ailments. The tribal communities depend on therapeutic plants because of their efficacy, lack of basic medical care facilities, and ethnic preferences [5]. The medicinal plants used in traditional remedies are mostly collected from the wild. Tribal people have diverse knowledge of traditional medicine based on local plants for basic medical care [6]. In tribal communities, traditional healers possess a lot of information about medicinal plants. In these regions, medicinal plants are important for the indigenous people, providing access to basic healthcare [7]. The traditional medicinal system acts as the principal supplier of primary healthcare services in the tribal areas because of the lack of modern healthcare facilities, the remoteness of the region, and a strong cultural belief in the efficacy of folk medicines [8].

The use of medicinal plants in everyday life has a long history and still has immense importance in aboriginal civilization [9]. In remote areas, therapeutic plants still play an important role [10] and are still used as the basic healthcare system. According to the literature, more than 50,000 flowering taxa have been used for medical purposes all over the globe [11]. Pakistan has diverse flora comprised of about 6000 flowering plant species [12, 13] and about 600 plant species have been identified with medicinal values [14]. About 80% of the inhabitants of remote areas of Pakistan are still dependent on medicinal plants [15]. Plant-derived medicines account for about 25% of all medicines available in the modern pharmacies, with many more artificial compounds isolated from plants.

In Pakistan, rural women frequently experience gynaecological disorders due to malnutrition, poor living standards, and hard physical work during pregnancy. A local woman, who is locally called “Dayiah,” is found in each village and specializes in herbal therapy to relieve gynaecological disorders with local medicinal plants [16]. The highest use of the therapeutic plant in rural communities is due to the high price of allopathic medicine and its side effects [17]. A traditional way of life, as well as a lack of a suitable approach to modern health facilities, motivates rural women to consult with nearby midwives and indigenous healers [18].

There is very limited literature on ethnogynaecology [19], whereas many reports on ethnobotanical and ethnomedicinal knowledge are available across the globe [18, 20]. Some ethnomedicinal surveys have been conducted to study the role of herbal therapy in women's medical and reproductive health disorders [20, 21]. Similarly, little literature is available about medicinal plants used by pastoral women for the healing of gynaecological problems. There is very little work carried out in Pakistan and in the whole world [22, 23]. Moreover, due to modernization and the lack of interest of younger generations in indigenous knowledge, which is declining speedily, ethnoecological information may vanish if not properly recorded [24]. In today's society, allopathic medicines, anti-inflammatory medicines, surgery, and nonsteroidal analgesics are commonly used to treat gynaecological disorders. These remedies are effective but usually have side effects, particularly when medicines are used for a long time. Moreover, some medicines used during the entire pregnancy period can harm the embryo [20].

This study aimed to record different types of plant species used against various gynaecological problems encountered by the female inhabitants of the tribal district of North Waziristan, Pakistan. The area is dominated by the Wazir and Dawar tribes, with low financial status, poor infrastructure, no modern medical facilities, and a lack of modern resources [14]. Many women and men in the region seek healing from a traditional therapist for a variety of problems related to the female reproductive organs. Such traditional knowledge has not been reported before from the study area as no ethnoecological documentation has been done earlier. Hence, this survey aims to report the ethnomedicinal knowledge of indigenous herbal remedies for the cure of gynaecological disorders and to preserve this precious but fast-vanishing indigenous knowledge of the tribal communities of the study area.

## 2. Methods

### 2.1. Study Area

Tribal district North Waziristan, Khyber Pakhtunkhwa, Pakistan, is the hilly region that lies between 32°35′ and 33°20′ north latitudes and 69°25′ and 70°40′ east longitudes, with an altitude of 2143–7717 feet. North Waziristan falls under the Irano-Turanian Region [25]. The area is bounded by mountains that are connected with Koh-e-Sulaiman in the south and Koh-e-Sufaid in the north. North Waziristan is bounded on the south by the district of South Waziristan; on the north by Kurram Agency, Hangu district, and Afghanistan; on the east by the district of Bannu; and on the west also by Afghanistan (Figure 1). The area is fertile and is irrigated by 3 rivers, namely, the Tochi, Kurram, and Katu rivers. The annual rainfall is 45 cm. The North Waziristan area contains 4,707 square kilometers (1,817 sq mi). There are two major tribes in the study area, that is, Wazir and Dawar. Pushto is the major language. The study area is one of the major war-affected areas of Pakistan. The total population in the conflict-affected area of North Waziristan is approximately 840,000. The region has been targeted with shelling and air raids, and at least 456,000 people, including nearly 200,000 children (42%), fled ahead of or during the ground assaults to safer parts of Pakistan and neighbouring Afghanistan.

### 2.2. Field Surveys and Medicinal Plants' Collection

The ethnogynaecological surveys were carried out in the tribal district (North Waziristan) from April 2018 to October 2020. Medicinal plants were collected during field visits [26, 27]. A collection number was given to each plant specimen with the help of tags. Plants were serially tagged and appropriately placed in the field presser. Snapshots of the collected plants were also captured [28, 29].

### 2.3. Questionnaires and Interviews

A semistructured questionnaire was used to collect the information regarding indigenous knowledge from the local informants and Hakeems of the study area [30–32]. Preference was given to elderly people and Hakeems. The collected specimens and photographs were further used in the interviews to recheck the information with other informants as well [28, 29]. A total of 130 local informants were interviewed, belonging to different age groups (35 years to 65 years), of which 105 were male and 25 were female, including housewives (daei/midwives and traditional healers) (Table 1) [33]. During the survey, local names, botanical names, folk uses, used parts, mode of preparation, mode of application (e.g., juice, paste, decoction, infusion, and powder), and growth/life form were documented by the local people of the study area. Through semistructured interviews [34, 35], knowledge about gender and age differences and occupation background and information about the herbal recipes for gynaecological disorders were documented [36].

### 2.4. Plant Identification and Preservation

The plant taxonomist Dr. Rahmatullah Qureshi identified the herbarium specimens and confirmed them with the help of available published literature [37]. These will be compared with identified specimens in the Herbarium of Pakistan Islamabad (ISL), Quaid-e-Azam University Islamabad. Medicinal plant species were also photographed at the time of collection [38, 39]. The collected plants' specimens were dried, pressed, poisoned with 1% HgCl_2_ solution, and mounted on standard-sized herbarium sheets (11.5 × 17.5 inch). A voucher number was assigned and the voucher specimens were submitted to the herbarium of the Department of Botany, Hazara University, Mansehra, Pakistan, for future references.

### 2.5. Quantitative Data Analysis

Indigenous knowledge is quantitatively analyzed using different quantitative indices [40–42] such as relative frequency of citation (RFC), used reports (UR), use value (UV), informant consensus factor (ICF), consensus index (CI%), fidelity level (FL%), and family importance value (FIV).

#### 2.5.1. Relative Frequency of Citation (RFC)

The RFC value for indigenous therapeutic plants is based on the number of informants for each plant species. A relative frequency of citation (RFC) is obtained by dividing the frequency of citation (FC) by the total number of informants in the survey (N). RFC was calculated by using the following formula [43, 44]:

(1) $$\begin{array}{c} \text{RFC}=\frac{FC}{N}\left(0<\text{RFC}<1\right), \end{array}$$

where FC is frequency of citation and *N* is total number of informants taking part in the survey (*N* = 130).

#### 2.5.2. Use Value (UV)

Use value (UV) of a species was determined by the following formula [45]:

(2) $$\begin{array}{c} \text{UV}=\frac{U}{n}, \end{array}$$

where *U* is number of use reports documented by the informants for a given medicinal plant and *n* is total number of informants interviewed for a specific medicinal plant.

#### 2.5.3. Consensus Index (CI%)

The percentage of local informants regarding their indigenous knowledge of therapeutic plants used to treat gynaecological problems was calculated by consensus index (CI%) [31]. The following formula was used:

(3) $$\begin{array}{c} \text{CI}=\frac{n}{N}\times 100, \end{array}$$

where “*n*” is the number of informants citing the medicinal plant species and “*N*” is the total number of respondents for the species during the survey.

#### 2.5.4. Fidelity Level (FL%)

The fidelity level (FL) is the percentage of informants who mention the utilization of particular medicinal plant species to cure specific ailments in the study area. The fidelity level (FL) is calculated by the following formula [46]:

(4) $$\begin{array}{c} \text{FL}\left(\%\right)=\frac{Np}{N}\times 100, \end{array}$$

where “*Np*” is the particular number of citations for a specific disease and “*N*” is the total number of respondents citing the plant species for any ailments.

#### 2.5.5. Informant Consensus Factor (ICF)

Informant consensus factor (ICF) was used to determine the informants' agreement on the reported treatment for any diseases group or ailment category [47]. The ICF value ranges from 0 to 1. Thus, the following formula was used:

(5) $$\begin{array}{c} \text{ICF}=\frac{\text{Nur}-Nt}{\text{Nur}}\mathrm{-1,} \end{array}$$

where Nur is the number of useful reports in any disease category and *Nt* is the number of plant species used.

#### 2.5.6. Family Importance Value (FIV)

To determine the importance of a family, the family importance value (FIV) was applied [44] using the following formula:

(6) $$\begin{array}{c} \text{FIV}=\frac{\text{FC}\left(\text{family}\right)}{N}\times 100, \end{array}$$

where FC is number of informants mentioning the family and *N* is total number of informants taking part in the survey (*N* = 130).

## 3. Results and Discussion

### 3.1. Informants' Demography

This study was conducted in the tribal district of North Waziristan, Pakistan. Inhabitants use medicinal plants for the cure of different gynaecological disorders. Demographic knowledge was acquired from the gender, age, education level, and practice of the informants. A total of 130 informants were interviewed, including 80.77% male and 19.23% female (Dayiahs). All the informants spoke Pushto. The dominance of male informants in the study area was greater as compared to females. There were certain cultural barriers due to which female informants could not talk with male interviewers outside of their families, but the investigated female informants gave their assent. Many of them were over 65 years old (47.69%), followed by 50–65 years old (40.77%) and 35–50 years old (11.54%). Participants were 76 herbalists, 29 professionals, and 25 housewives (Table 1). The majority of herbal healers in this study were males. These results are similar to the previous literature [48]. Based on educational facilities, the indigenous knowledge and use of therapeutic plants for the treatment of gynaecological disorders were more prevalent in the illiterate people, that is, 40.77%, and the same traditional knowledge was declining in the graduate level (5.38%) of the study area. Based on age, it was observed that the indigenous knowledge and use of medicinal plants remedies for gynaecological disorders were more prevalent in the elders. The same results were documented by other authors from nearby areas and other countries [49, 50]. The inherited traditional knowledge of therapeutic plants is transferred orally and verbally from their ancestors and passed from generation to another [24]. Noticeably, information and knowledge related to the traditional medication of gynaecological disorders are vanishing due to the death of older females (Dayiahs) in the community. Hence, there is a dire need to conserve this indigenous knowledge from extinction [5].

### 3.2. Indigenous Medicinal Plants' Diversity

The study area has a wealthy floral diversity. For their basic medical care needs, tribal people have varying knowledge of traditional medicine associated with medicinal plants. All medicinal plant species along with their qualitative analysis (botanical names, family name, parts used, mode of preparation, mode of application, and disease treated) and quantitative analysis (RFC, FL, ICF, UV, and UR) of each medicinal plant species were calculated and are presented in Table 2. In this study, 67 medicinal plants belonging to 38 families were recorded as being used to treat gynaecological disorders by the indigenous people of tribal district of North Waziristan, Pakistan. Approximately, 84% of the rural population depends on herbal therapeutic plants [51]. In rural areas of Pakistan, approximately 75% of the inhabitants are still reliant on traditional knowledge for their basic healthcare system [52], because there is no modern healthcare facility provided to them. Thus, most of the inhabitants are dependent on herbal remedies in the study area. The most dominant family was the Lamiaceae with 7 species, followed by Asteraceae and Rosaceae with 4 species each (Table 2). The family Lamiaceae is predominant in the study area similar to the results reported in the previous work [53].

### 3.3. Life Form of the Ethnomedicinal Flora

In terms of life forms, the most dominant life form used in gynaecological remedies was herbs (42 species, 62.69%), followed by shrubs (15 species, 22.39%), trees (7 species, 10.45%), ferns (2 species, 2.99%), and sedge (1 species, 1.49%) (Figure 2). The frequent use of herbs in herbal remedies has also been documented in other areas of the globe [54, 55]. Herbs often have a high content of bioactive compounds [56], are easily accessible, and have profuse growth in wild varieties. Similar to other studies carried out by [57], easy accessibility of herbaceous plants or therapeutic plants, valuable healing action, and reasonable cost of the healthcare system are the major factors for the preference and advancement of herbal medication in the economically backward rural communities [58].

### 3.4. Plant Parts Used in Herbal Remedies

Various plant parts are regarded as useful in various ailments. The indigenous communities of North Waziristan, Pakistan, use approximately all parts of the medicinal plants as remedies for gynaecological problems. The most highly utilized parts for herbal remedies observed were leaves (16 species, 22.54%), followed by the whole plant (15 species, 21.13%), roots (12 species, 16.90%), seed (7 species, 9.86%), fruits (6 species, 8.45%), aerial parts, gum and shoots (3 species, 4.23% each), bark and bulb (2 species, 2.82% each), and flower and rhizome (1 species, 1.41% each) (Figure 3). The collection of leaves and medication preparation from leaves are so easy as compared to the other plant parts. For these purposes, leaves are commonly used in folk remedies [59]. The removal of leaves from the medicinal plants can cause less harm as compared to the removal of other parts of the plant [60]. The high use of leaves in herbal remedies preparation is also reported in other study areas [61–63].

### 3.5. Preparation of Remedies

Medicinal plants were used by the indigenous people in diverse ways and in various recipes. A total of 14 modes of preparation were used in the indigenous communities. In the current study, decoction (25 species, 36.76%) is the dominant methodology used for the preparation of herbal remedies, followed by powder (22 species, 32.35%), juice (4 species, 5.88%), paste (3 species, 4.42%), herbal tea, poultice, raw, and smoke (2 species, 2.94% each) (Figure 4). Similarly, decoction and powder were reported as the most commonly used methods for preparing herbal remedies in other studies [64, 65].

### 3.6. Mode of Administration

In this study, the dominant modes of administration/application were orally advised (62 species, 92.54%), followed by inhaling and topical (2 species, 92.54% each), and chewing (1 species, 1.49%) (Figure 5). The majority of oral administration was also reported in other study areas [66, 67].

### 3.7. Indigenous Plants Used for the Treatment of Gynaecological Disorders

Tribal people have a wide range of knowledge about traditional medicine based on local plants for basic medical care [6]. During this ethnogynaecological study, 26 gynaecological disorders were documented, which were treated by using 67 medicinal plants (Table 3). The common gynaecological disorder in the study area was irregular menstrual flow, which was treated by using 11 plant species (15.28%), followed by leucorrhoea (8 species, 11.11%), enhanced milk flow and gonorrhea (6 species, 8.33% each), excessive menstruation (4 species, 5.56%), abnormal stoppage of menstruation, abortion, easy delivery, miscarriage, and vomiting (3 species, 4.17% each).

### 3.8. Quantitative Analysis

The recorded data were analyzed through different statistical indices like RFC, UV, CI%, ICF, FL%, and FIV.

#### 3.8.1. Relative Frequency of Citation (RFC)

A relative frequency of citation was used to assess the most commonly used therapeutic plants [68] for gynaecological disorders. In this study, the RFC ranged from 0.11 to 0.37 (Table 2). Based on RFC values, the most valuable medicinal plant having a high degree of RFC was *Acacia modesta* (0.37), followed by *Cydonia oblonga* (0.36), *Berberis lycium, Tecomella undulata, Trianthema portulacastrum,* and *Withania somnifera* (0.35). The lowest RFC value was calculated for *Ajuga parviflora* (0.11). Those therapeutic plant species having the highest RFC value should be further analyzed pharmaceutically and phytochemically to identify their bioactive compounds for medicinal discovery [69, 70].

#### 3.8.2. Use Value (UV)

According to [45], the use value indexation is a quantitative technique of ethnobotany that correlates the importance of plant species among aboriginal communities with regard to their uses. The use value in our documented data ranged from 0.27 to 0.85 and the use reports (URs) ranged from 9 to 39 (Table 2). The highest use value was reported for *Tecomella undulata* (0.85), followed by *Cydonia oblonga* (0.81), *Withania somnifera* (0.78), *Acacia modesta* (0.77), and *Berberis lycium* (0.76). The lowest use value (UV) was recorded for *Cyperus rotundus* (0.27). It was observed that the maximum use values were due to the higher number of use reports (URs) in the study area. The highest used values of documented therapeutic plants might indicate their indigenous professional expertise, which leads to a preference option for the disorder [71]. Medicinal plants with the lowest UV do not mean that they are not medicinally important, but it is shown that the traditional knowledge about these medicinal plants is limited [72]. Therapeutic plants for which the use value (UV) is high due to their frequent distribution in the research area and the inhabitants are well known for their medicinal value [35].

#### 3.8.3. Consensus Index (CI%)

The percentage of informants having traditional indigenous knowledge of medicinal plant species used for illness control (in this study, gynaecological disorders) was determined using a consensus index (CI%) [73], which indicates the citation by percent of informants [74]. The consensus index (CI) value ranges from 10.77% to 36.92% (Table 2). The maximum CI value was obtained for *Acacia modesta* (36.92%), followed by *Cydonia oblonga* (36.15%), *Tecomella undulata,* and *Withania somnifera* (35.38%). The lowest consensus index (CI) value was calculated for *Ajuga parviflora* (10.77%). CI indicates an agreement on the fact that *Acacia modesta* and *Cydonia oblonga* are the most important and well-known therapeutic plants used for the treatment of gynaecological disorders in North Waziristan.

#### 3.8.4. Fidelity Level (FL%)

Fidelity level (FL%) is used to determine the medicinal plant species that are most preferred by indigenous people for the cure of any specific ailment [46]. The therapeutic plants with the highest healing effects have the maximum fidelity level of 100%. The medicinal plant species that were mentioned by a single informant were not considered for the FL level study. In this study, FL ranged from 44.44% to 100% (Table 2). It is a fact that the higher the plant's utilization is, the higher the FL value will be. In this study, the highest FL was determined for *Acacia modesta* (backache after delivery), *Berberis lycium* (gonorrhea), and *Cydonia oblonga* (leucorrhoea) (100%), followed by *Carum carvi* (97.73%) for expelling impurities from the uterus and *Tamarix aphylla* (95.24%) for antiseptic, while the lowest FL was recorded for *Convolvulus arvensis* (44.44%) for irregular menstrual flow. The highest value of fidelity level (FL) determined the choice of informants to cure the specific disease [75].

#### 3.8.5. Informant Consensus Factor (ICF)

The informant consensus factor (ICF) establishes the even sharing of informants' information regarding the medicinal plants, which validates that all the local people in the research area use plants for the treatment of the same ailment in same or different methods. In other words, the ICF value explains the cultural consistency in the use of a group of medicinal plants to treat a specific ailment [76]. To determine the informants' consensus factor (ICF), various diseases were grouped into 14 different disease categories based on taxa and use reports (Table 4). In this study, the ICF values ranged from 0.96 to 1.0. The highest ICF value was reported for emmenagogue and tonic after delivery (1.0), followed by antiseptic (0.99), and the lowest ICF value was reported for menstrual problems (0.96). Similar results were reported by [77] demonstrating that emmenagogue disorder has the highest ICF values.

#### 3.8.6. Family Importance Value (FIV)

The family importance value increases with the increase in the frequency of citations of all species. In this work, the most important family, based on the frequency of citations, was Lamiaceae with an FIV value of 98.46%, followed by Rosaceae (93.85%), Apiaceae (86.92%), Solanaceae (86.15%), Asteraceae (76.92%), and Mimosaceae (75.38%). Convolvulaceae has the lowest family importance value, with 13.85% (Table 5). Medicinally important plant species of the families Asteraceae, Apiaceae, Lamiaceae, and Rosaceae are mentioned as important in various pharmacological works [78, 79]. The highest FIV value percentage reveals that the plants of a specific family are commonly used in treating various disorders, as reported by informants.

### 3.9. Status of Medicinal Plants

According to local residents, the population of most medicinal plants has decreased over the last few decades. Threatened and endangered species of the study area are *Berberis lycium*, *Fritillaria imperialis*, *Gymnosporia nemorosa*, *Pistacia integerrima*, and *Tecomella undulata*. Excessive and injudicious use, overgrazing, improper harvesting practices such as digging out the entire plant, market pressure, and deforestation are also contributing factors. Medicinal plants are collected from the study area, transported to a small market by locals, and then exported to major cities. Locals also use shrubby species and trees as fuel sources, which have a negative impact on medicinal plant populations. Forests are necessary for the survival of several therapeutic plant species. As a result, the area's medicinally important plants are decreasing. Such flora need preservation through sustainable use, appropriate management, and conservation. A regional awareness campaign regarding the state of indigenous flora, sustainable plant harvesting, and the conservation of valuable therapeutic plants will lead to better outcomes. Local inhabitants, local stakeholders, and plant collectors should be aware of the conservation of plant resources in the region, and the indigenous people should be involved in conservation practices.

### 3.10. Novelty and Future Impacts

This study was compared with previously published literature of neighbouring areas and distant areas of utilization of medicinal plants for ethnogynaecological disorders [18, 80–86]. The comparative study between previously reported medicinal plants showed that some medicinal plants have the same or different medicinal uses, while some were documented for the first time and others were not previously documented. The following 9 species were reported for the first time to cure gynaecological diseases: *Acacia modesta* (aphrodisiac), *Cnicus benedictus* (enhance milk flow)*, Cocculus pendulus* (amenorrhea)*, Cydonia oblonga* (leucorrhoea)*, Cyperus rotundus* (enhance milk flow), *Peganum harmala* (antiseptic)*, Prunus domestica* (vomiting)*, Tamarix aphylla* (antiseptic), and *Tecomella undulata* (leucorrhoea) (Table 2). Many ethnomedicinal studies have similar medicinal uses of therapeutic plants for the treatment of various ailments all over the globe. This study adds some new therapeutic plant uses, which may provide baseline data for phytochemical and pharmacological screening for the detection of new drugs in future studies. The discovery of drugs from therapeutic plants links an interdisciplinary approach to joining ethnomedicinal, pharmacological, botanical, and natural methods. However, any medicinal plants in this study area are not subjected to detailed pharmacological screenings.

## 4. Conclusion

This study focuses on pastoral women's health and healing. In rural areas, modern health facilities are insufficient or not available. Rural people (midwives, traditional healers) have indigenous knowledge of herbal remedies for treating gynaecological disorders. In the research area, 67 therapeutic plants are used to treat 26 different types of gynaecological disorders. Leaves are the dominant part used in the preparation of herbal remedies for gynaecological disorders. Menstrual problems were the most prevalent ailment category treated using 26 therapeutic plants in the study area. Decoction and powder were reported as the most commonly used methods for preparing herbal remedies, which clearly shows the consistency with other studies as well [53, 54]. The highest use value was reported for *Tecomella undulata* (0.85), followed by *Cydonia oblonga* (0.81) and *Withania somnifera* (0.78). It was observed that the medicinal plants having maximum UV were due to their higher number of use reports (URs) in the study area. The literature reveals that the therapeutic plants with higher UV are because of their frequent distribution in the research area and the inhabitants are well known for their medicinal value [62], which leads them to be the preferred option for the particular ailment [59]. The cultural consistency in the use of a group of medicinal plants to treat a specific ailment group was explained using ICF [47], through which the consistency of our results was found in accordance with Sadeghi et al. [20]; they reported that emmenagogue disorder has the highest ICF values. Some medicinal plants, like *Berberis lycium*, *Fritillaria imperialis*, *Gymnosporia nemorosa*, *Pistacia integerrima*, and *Tecomella undulata* are under extreme pressure as a result of the indiscriminate collection by locals. We believe that forest protection and floral habitat conservation are critical. For this, the government and nongovernmental organizations (NGOs) must design appropriate programmes with the participation of local people who must be educated about the need to maintain precious forest resources and participate in forestation for future generations. This survey provides a baseline for future clinical and pharmacological studies in the field of gynecology. Therefore, it is necessary to focus on the medicinal uses of the reported plants [48]. Detailed clinical and pharmacological trials are needed to find out the bioactive components for the treatment of the gynaecological disorder.

## Figures and Tables

**Figure 1:** Map of the study area (North Waziristan, KP, Pakistan). The black dots indicate the visited sites for the study.

**Figure 2:** The proportion of various plant life forms.

**Figure 3:** Plant parts are used in herbal remedies. The blue bar shows the “number of species.”

**Figure 4:** Mode of herbal drug preparation. The blue bar shows the “number of species.”

**Figure 5:** Mode of application/administration. The blue bar shows the “number of species.”

**Table 1:** Demographic information of the Informants.

Variable	Categories	No. of informants *N* = 130	Percentage (%)
Gender	Male	105	80.77
	Female (Dayiahs/midwives)	25	19.23

Informant category	Traditional healers	90	69.23
	Indigenous people	40	30.77

Occupation	Herbalists	76	58.46
	Housewives	25	19.23
	Professional	29	22.31

Age	35–50	15	11.54
	50–65	53	40.77
	Above 65	62	47.69

Education level	Illiterate	53	40.77
	Primary level	34	26.15
	Middle level	15	11.54
	Secondary level	12	09.23
	Undergraduate (Hakims)	9	06.92
	Graduate (Hakims)	7	05.38

**Table 2:** Medicinal plants with the quantitative analysis used for gynaecological disorders by the local communities of the tribal district of North Waziristan, Pakistan.

Plants species	Family name	Vernacular name	Voucher no.	Habit	Parts used	Mode of preparation	Gynaecological use	Mode of application	FC	RFC	UR	UV	CI%	FL%
*Abutilon indicum* (L.) Sweet	Malvaceae	Zergulai	SR-13340	Shrub	Root	Powder + honey + milk	Leucorrhoea	The mixture of about one glass is taken once a day for seven days for the treatment of leucorrhoea.	40	0.31	20	0.50	30.77	57.50
*Acacia modesta* Wall.	Mimosaceae	Palusa	SR-13196	Tree	Gum	Powder + butter oil + milk	Backache after delivery, aphrodisiac	The mixture of about one cup is taken twice a day for 3–5 days to treat backache after delivery and used as an aphrodisiac.	48	0.37	37	0.77	36.92	100.00
*Acacia nilotica* (L.) Willd. ex Delile	Mimosaceae	Kekar	SR-13448	Tree	Bark	Decoction	Gonorrhea	Decoction of one medium size cup is taken for three days to cure gonorrhea.	27	0.21	14	0.52	20.77	62.96
*Achyranthes aspera* L.	Amaranthaceae	Ghoshkai	SR-13311	Herb	Leaves	Decoction	Labour pain	Decoction of leaves (half cup) is used to reduce excessive labour pain.	23	0.18	12	0.52	17.69	69.57
*Adiantum capillus-veneris* L.	Adiantaceae	Ebe betai	SR-13459	Ferns	Leaves	Decoction	Abnormal stoppage of menstruation	Decoction of leaves of about one medium size cup for 4-5 days is taken and used as menstruation additive.	24	0.18	16	0.67	18.46	50.00
*Ajuga bracteosa* Wall.	Lamiaceae	Varekai boti	SR-13425	Herb	Whole plant	Decoction	Abnormal stoppage of menstruation	Decoction of aerial parts of about 1 cup for three days is taken and used as menstruation additive.	20	0.15	13	0.65	15.38	55.00
*Ajuga parviflora* Benth.	Lamiaceae	Shengulai	SR-13413	Herb	Leaves, roots	Powder + milk	Amenorrhea	Powder (3 tablespoons) is given with one glass of warm milk for 6-7 days used to cure amenorrhea.	14	0.11	8	0.57	10.77	50.00
*Allium sativum* L.	Alliaceae	Yeza	SR-13462	Herb	Bulb	Powder + curcumin powder	Easy delivery	Powder of 2 : 1 spoons is given to pregnant women with one glass of water used to stimulate uterine muscles for easy delivery.	25	0.19	13	0.52	19.23	56.00
*Amaranthus spinosus* L.	Amaranthaceae	Geta pakhe	SR-13326	Herb	Roots	Decoction	Excessive menstruation	Decoction of roots (one cup) is taken for 3 days and used to reduce menstrual flow.	21	0.16	11	0.52	16.15	57.14
*Amaranthus viridis* L.	Amaranthaceae	Surme	SR-13341	Herb	Leaves	Paste	Leucorrhoea	Leaves are cooked in oil and jaggery (gur) and the paste is taken for five days to treat leucorrhoea.	22	0.17	13	0.59	16.92	59.09
*Androsace rotundifolia* Hardw.	Primulaceae	Sergulai	SR-13424	Herb	Leaves	Juice	Irregular menstrual flow	Fresh juice (2 spoons) for 5–7 days is taken to regularize menstrual flow.	26	0.20	9	0.35	20.00	61.54
*Berberis lycium* Royle	Berberidaceae	Therkha	SR-13444	Shrub	Roots	Decoction	Gonorrhea	Decoction of roots (2 spoons) is taken for 7–10 days to cure gonorrhea.	45	0.35	34	0.76	34.62	100.00
*Boerhavia diffusa* L.	Nyctaginaceae	Pret boti	SR-13373	Herb	Aerial parts	Decoction	Irregular menstrual flow	Decoction of aerial parts (1 spoonful) is given twice a day for seven days to regularize menstrual flow.	39	0.30	28	0.72	30.00	61.54
*Bupleurum falcatum* L.	Apiaceae	Pest boti	SR-13443	Herb	Whole plant	Decoction	Irregular menstrual flow	Decoction of the whole plant (3 spoons) is taken once a day for fifteen days to regulate the menses.	28	0.22	13	0.46	21.54	64.29
*Calendula arvensis* M.Bieb.	Asteraceae	Zer gulai	SR-13367	Herb	Flower	Infusion	Painful menstruation	Infusion of flowers (10–15 ml) is taken twice a day to cure pain during menstruation.	25	0.19	10	0.40	19.23	48.00
*Capsella bursa-pastoris* (L.) Medik.	Brassicaceae	Push boti	SR-13477	Herb	Aerial parts	Decoction	Irregular menstrual flow	Decoction of aerial pats (2 spoonful) is taken thrice a day for 3–5 days to regularize menstrual flow.	34	0.26	12	0.35	26.15	50.00
*Carum carvi* L.	Apiaceae	Zera	SR-13467	Herb	Seeds	Powder + butter oil	Expel impurities from the uterus	Powder of seeds (10 g) is mixed with butter oil, taken once a day for 5 days, and used to expel impurities from the uterus.	44	0.34	31	0.70	33.85	97.73
*Chenopodium ambrosioides* L.	Chenopodiaceae	Khersapaka	SR-13531	Herb	Leaves	Decoction	Painful menstruation, enhance milk flow	Leaves decoction (one cup) given twice a day for three days is recommended for painful menstruation. The same is given to nursing mothers to enhance the flow of breast milk.	41	0.32	27	0.66	31.54	56.10
*Citrullus colocynthis* (L.) Schrad	Cucurbitaceae	Maraginye	SR-13486	Herb	Fruit	Juice	Easy delivery	Fresh juice of fruit (two spoons) is given to women during childbirth and is used for easy and smooth delivery.	39	0.30	21	0.54	30.00	71.79
*Cnicus benedictus* L.	Asteraceae	Pest azghi	SR-13473	Herb	Aerial parts	Decoction + milk	Enhance milk flow	A decoction of aerial parts (one spoonful) is mixed with one glass of milk and given to nursing mothers to increase the flow of breast milk.	27	0.21	14	0.52	20.77	77.78
*Cocculus pendulus* (J.R. Forst. and G. Forst.)	Menispermaceae	Motiki boti	SR-13573	Shrub	Roots	Decoction	Amenorrhea	Decoction of roots (15 ml) is given for 7–10 days continuously to treat amenorrhea.	43	0.33	31	0.72	33.08	53.49
*Convolvulus arvensis* L.	Convolvulaceae	Pervetia	SR-13215	Herb	Whole plant	Decoction	Irregular menstrual flow	Decoction of the plant (4 tea spoonful) is taken for 3-4 days to regulate menstrual flow.	18	0.14	10	0.56	13.85	44.44
*Cydonia oblonga* Mill.	Rosaceae	Bahi	SR-13520	Shrub	Fruit, seeds	Jame, powder	Nausea and vomiting, leucorrhoea	Fruit jam (two teaspoonful) is given to pregnant women once in the early morning on an empty stomach for 3 days to treat nausea and vomiting. Seeds powder (1 teaspoonful) is mixed with honey and given once a day for 7 days to treat leucorrhoea.	47	0.36	38	0.81	36.15	100.00
*Cyperus rotundus* L. K	Cyperaceae	Delgai	SR-13296	Sedge	Rhizome	Poultice	Enhance milk flow	A poultice of the rhizome is applied to the breast to increase the flow of breast milk.	33	0.25	9	0.27	25.38	63.64
*Datura stramonium* L.	Solanaceae	Berbaka	SR-13376	Shrub	Leaves	Poultice	Breast swelling	A poultice of fresh leaves is topically applied on a nursing mother's breast to cure the inflammation of breasts.	23	0.18	12	0.52	17.69	82.61
*Dodonaea viscosa* (L.) Jacq	Sapindaceae	Ghavajara	SR-13269	Shrub	Leaves	Decoction	Excessive menstruation	Decoction of leaves (two spoons) is taken twice a day for 3 days to control excessive menstruation.	43	0.33	27	0.63	33.08	79.07
*Eclipta prostrate* (L.)	Asteraceae	Thorkvanai	SR-13359	Herb	Whole plant	Herbal tea	Miscarriage	Herbal tea (1 tea spoonful) is given twice a day for 7 days to prevent miscarriage.	23	0.18	12	0.52	17.69	73.91
*Equisetum arvense* L.	Equisetaceae	Bandkai	SR-13216	Ferns	Whole plant	Decoction	Gonorrhea	Decoction of plant (15–20 ml) is given once a day for 4-5 days and used to cure gonorrhea.	27	0.21	13	0.48	20.77	77.78
*Erodium cicutarium *L.	Geraniaceae	Not known	SR-13209	Herb	Whole plant	Herbal tea + jaggery	Irregular menstrual flow, enhance milk flow	Herbal tea (two teaspoonful) with jaggery is given twice a day to regulate menstrual flow. The same is given to nursing mothers to increase the flow of breast milk.	33	0.25	19	0.58	25.38	72.73
*Euphorbia hirta* L.	Euphorbiaceae	Bayavenia	SR-13529	Herb	Whole plant	Latex	Enhance milk flow	Latex (10 ml) is given once a day to the nursing mother to increase the flow of breast milk.	31	0.24	16	0.52	23.85	70.97
*Fragaria nubicola* (Hook.f.) Lindl.	Rosaceae	Jangli strawberi	SR-13429	Herb	Fruit	Raw	Irregular menstrual flow	Fruits (5–10) are taken twice a day for three days to regulate menstrual flow.	25	0.19	8	0.32	19.23	64.00
*Fritillaria imperialis* L.	Liliaceae	Geger Gul	SR-13383	Herb	Bulb	Powder + milk	Enhance milk flow	Bulb powder (one spoon) is given with one cup of milk to nursing mothers once a day for 7 days to increase the flow of breast milk.	25	0.19	11	0.44	19.23	52.00
*Geranium wallichianum* D. Don ex sweet	Geraniaceae	Varekai bote	SR-13389	Herb	Roots	Powder + milk	Leucorrhoea, tonic after delivery	Roots powder (1 teaspoonful) mixed with milk and sugar is given twice a day for 3–5 days to cure leucorrhoea and is also used as tonic after delivery.	41	0.32	23	0.56	31.54	78.05
*Gymnosporia nemorosa* (Eckl. & Zeyh.) Szyszyl.	Celastraceae	Sagherzai	SR-13364	Shrub	Fruit	Powder + butter oil	Labour pain	Fruit powder (10–12 gm) mixed with butter oil is given to pregnant women during childbirth to reduce excessive labor pain.	29	0.22	11	0.38	22.31	72.41
*Justicia adhatoda* L. K	Acanthaceae	Bikarh	SR-13233	Shrub	Root, leaves	Paste + milk	Leucorrhoea	Roots paste (2 teaspoonful) mixed with one glass of milk is given twice a day for 15 days of and used to cure leucorrhoea.	33	0.25	16	0.48	25.38	66.67
*Lepidium sativum* L.	Brassicaceae	Bashke	SR-13320	Herb	Seeds	Powder + milk	Abnormal stoppage of menstruation	Seeds powder (5-6 g) mixed with one glass of milk is given once a day for 3–5 days and used as a menstruation additive.	20	0.15	9	0.45	15.38	65.00
*Leucaena leucocephala* (Lam.) de Wit	Mimosaceae	Pest kekar	SR-13358	Shrub	Seeds	Powder + honey	Menstrual cramps	Seeds powder (10 g) mixed with honey and taken twice a day for 4-5 days is recommended for menstrual cramps.	23	0.18	11	0.48	17.69	60.87
*Melia azedarach* L.	Meliaceae	Bakana	SR-13266	Tree	Fruit gum	Powder + cow's milk	Emmenagogue	Fruits gum powder (4-5 g) mixed with cow's milk and given to women once a day for 2-3 days is recommended for emmenagogue.	44	0.34	27	0.61	33.85	70.45
*Mentha spicata* L.	Lamiaceae	Velanai	SR-13283	Herb	Leaves	Juice	Easy delivery	Juice of leaves (one glass) is given to expectant mother to speed up child birth.	20	0.15	13	0.65	15.38	65.00
*Mentha arvensis* L.	Lamiaceae	Sarkori Velanai	SR-13284	Herb	Whole plant	Powder	Antifertility	Powder of plant (2 spoons) mixed with one glass of water is given to women before the meeting and used for antifertility.	21	0.16	11	0.52	16.15	85.71
*Mirabilis jalapa* L.	Nyctaginaceae	Mazdergul	SR-13500	Herb	Roots	Powder + milk	Sexual tonic	Roots powder (1 spoonful) mixed with one glass of milk is taken during nighttime daily for 7 days and used as a sexual tonic.	36	0.28	16	0.44	27.69	80.56
*Nasturtium officinale* R.Br.	Brassicaceae	Mangore	SR-13317	Herb	Leaves, shoots	Juice	Produce temporary sterility	Juice of plant (one cup) is given to women daily for 3–5 days to produce temporary sterility.	28	0.22	14	0.50	21.54	78.57
*Nepeta cataria* L.	Lamiaceae	Khezbe	SR-13420	Herb	Whole plant	Decoction	Delayed menses	Decoction of plant (one cup) taken once a day for 5–7 days is recommended to delay menstruation.	18	0.14	10	0.56	13.85	72.22
*Opuntia dillenii* Haw.	Cactaceae	Sapre boti	SR-13168	Shrub	Fruit	Baking + honey	Gonorrhea	Fruit juice is baked and mixed with honey and given twice a day for 10 days to cure gonorrhea.	40	0.31	22	0.55	30.77	77.5
*Oxalis corniculata* L.	Oxalidaceae	Threw boti	SR-13254	Herb	Leaves	Chewing	Vomiting	The leaves are chewed to avoid vomiting during the early period of pregnancy.	37	0.28	19	0.51	28.46	59.46
*Peganum harmala* L.	Zygophyllaceae	Sponda	SR-13163	Herb	Whole plant	Smoke	Antiseptic	The smoke of the plant passed on to the women after childbirth is used as an antiseptic.	40	0.31	19	0.48	30.77	95.00
*Phyla nodiflora* (L.) Greene.	Verbenaceae	Ebe betai	SR-13319	Herb	Roots	Decoction + honey	Infertility	Decoction of root (10–12 ml) with honey (2 spoons) is given to women for promoting sexual desire.	16	0.12	8	0.50	12.31	50.00
*Pistacia integerrima* J. L. Stewart ex Brandis.	Anacardiaceae	Shene	SR-13464	Tree	Gum	Powder + milk	Gonorrhea	Gum powder (8 g) mixed with milk and sugar is given once a day for 12 days to cure gonorrhea.	43	0.33	21	0.49	33.08	90.70
*Portulaca oleracea* L.	Portulacaceae	Parkhorai	SR-13169	Herb	leaves	Cooked	Excessive menstruation	Leaves are cooked in oil and black pepper and this paste is given for 3-4 days to control excessive menstruation.	31	0.24	16	0.52	23.85	74.19
*Potentilla erecta* (L.) Raeusch.	Rosaceae	Dhania ghonde	SR.13432	Herb	Whole plant	Powder + curd	Excessive menstruation	Powder of plant (10 g) mixed with curd is taken daily for 3 days to control excessive menstruation.	25	0.19	11	0.44	19.23	60.00
*Prunus domestica* L.	Rosaceae	Manra	SR-13521	Tree	Fruit	Raw	Vomiting	The unripe fruit is given to pregnant women to avoid vomiting during the early period of pregnancy.	25	0.19	17	0.68	19.23	72.00
*Ricinus communis* L.	Euphorbiaceae	Arind	SR-13132	Shrub	Seed	Powder	Abortion	Powder of seeds (15–20 g) is given with water to pregnant women for 3 days at the initial stage to induce abortion.	37	0.28	18	0.49	28.46	72.97
*Solanum surattense* Burm. f.	Solanaceae	Kurkundai	SR-13396	Herb	Whole plant	Decoction + jaggery	Conception	Decoction of the plant (one cup) mixed with jaggery is given for 5 days to promote the chance of pregnancy in females.	43	0.33	27	0.63	33.08	90.70
*Tagetes erecta* L.	Asteraceae	Zenda gula	SR-13260	Herb	Roots	Decoction	Irregular menstruation	Decoction of roots (10–12 ml) is taken once a day for 3-4 days to regulate menstruation.	25	0.19	13	0.52	19.23	56.00
*Tamarix aphylla* (L.) H. Karst.	Tamaraceae	Ghaz	SR-13215	Tree	Leaves	Smoke	Antiseptic	The smoke passed on to women after childbirth is used as an antiseptic.	42	0.32	23	0.55	32.31	95.24
*Tecomella undulata* (Roxb.) Seeman.	Bignoniaceae	Rawdana	SR-13378	Shrub	Bark	Decoction + sugar	Lecucorroea	Decoction of the bark (one cup) mixed with sugar is given twice a day for 7 days to cure leucorrhoea.	46	0.35	39	0.85	35.38	97.83
*Teucrium stocksianum* Boiss.	Lamiaceae	Malgai	SR-13274	Herb	Shoots	Powder + milk	Conception, miscarriage	Powder of shoot (8–10 g) mixed with milk is taken once a day for 5 days to increase chances of fertilization and to prevent miscarriage.	20	0.15	11	0.55	15.38	90.00
*Thymus serpyllum* L.	Lamiaceae	Pestekai	SR-13451	Herb	Whole plant	Decoction + sugar	Irregular menstruation	Decoction of the plant (one cup) mixed with sugar is given once a day for 3-4 days to regulate menses.	15	0.12	8	0.53	11.54	60.oo
*Trachyspermum ammi* (L.) Sprague	Apiaceae	Sperkai	SR-13206	Herb	Seeds	Powder	Irregular menstruation	Powder of the seeds (15–20 g) is taken with water twice a day for 3-4 days to regulate menstruation.	41	0.32	21	0.51	31.54	95.12
*Trianthema portulacastrum* L.	Azoiaceae	Mardor betai	SR-13339	Herb	Whole plant	Decoction	Abortion	Decoction of the plant (one glass) is given twice a day to pregnant women in the early period of pregnancy to induce abortion.	45	0.35	27	0.60	34.62	77.78
*Tribulus terrestris* L.	Zygophyllaceae	Markhiri	SR-13236	Herb	Leaves	Decoction + sugar	Gonorrhea	Decoction of leaves (one cup) mixed with sugar is taken once a day for 5–7 days to cure gonorrhea.	17	0.13	9	0.53	13.08	88.24
*Urtica dioica* L.	Urticaceae	Sezankai	SR-13128	Herb	Whole plant	Powder + cow's milk	Leucorrhoea	Powder of the plant (12–15 g) mixed with one glass of cow's milk is taken twice a day for 15 days to cure leucorrhoea.	19	0.15	8	0.42	14.62	63.16
*Verbena officinalis* L.	Verbenaceae	Bachawai	SR-13293	Herb	Whole plant	Decoction	Miscarriage	Decoction of the plant (one cup) is given once a day for 5 days to prevent miscarriage.	23	0.18	11	0.48	17.69	60.87
*Vitex negundo* L.	Verbenaceae	Marwandai.	SR-13171	Shrub	Shoots	Decoction + honey	Irregular menstruation	Decoction of the shoots (two teaspoonful) mixed with honey is taken once a day for 3-4 days to regulate menstrual flow.	26	0.20	14	0.54	20.00	65.38
*Withania somnifera* (L.) Dunal	Solanaceae	Sre dane	SR-13230	Shrub	Roots	Powder + butter oil	Sexual tonic	Powder of roots (6–8 g) mixed with butter oil is taken once a day during nighttime for 10 days to stimulate sexual desire.	46	0.35	36	0.78	35.38	84.78
*Ziziphus mauritiana* Lam.	Rhamnaceae	Bara	SR-13198	Tree	Seeds	Paste	Leucorrhoea	The paste made from seeds is given twice a day for 15 days to cure leucorrhoea.	21	0.16	11	0.52	16.15	76.19
*Ziziphus nummularia* (Burm. f.) Wight and Arn.	Rhamnaceae	Karkana	SR-13179	Shrub	Roots	Powder	Abortion	Powder of the roots (8–10 g) is given with water twice a day to pregnant women in the early stage of pregnancy to induce abortion.	37	0.28	21	0.57	28.46	70.27

RFC: relative frequency of citation, FC: frequency of citation, UR: used reports, UV: use value, FL%: fidelity level, FIV: family importance value.

**Table 3:** Gynaecological diseases treated by using indigenous plants.

Sr. no.	Diseases	Number of species	Percentage
1	Abnormal stoppage of menstruation	3	4.17
2	Abortion	3	4.17
3	Amenorrhea	2	2.78
4	Antifertility	1	1.39
5	Antiseptic	2	2.78
6	Backache after delivery	1	1.39
7	Breast swelling	1	1.39
8	Conception	2	2.78
9	Delayed menses	1	1.39
10	Easy delivery	3	4.17
11	Emmenagogue	1	1.39
12	Enhance milk flow	6	8.33
13	Excessive menstruation	4	5.56
14	Expel impurities from uterus	1	1.39
15	Gonorrhea	6	8.33
16	Infertility	1	1.39
17	Irregular menstrual flow	11	15.28
18	Labour pain	2	2.78
19	Leucorrhoea	8	11.11
20	Menstrual cramps	1	1.39
21	Miscarriage	3	4.17
22	Painful menstruation	2	2.78
23	Produce temporary sterility	1	1.39
24	Sexual tonic	2	2.78
25	Tonic after delivery	1	1.39
26	Vomiting	3	4.17

**Table 4:** Informant consensus factor (ICF) value for various diseases categories.

Sr. no.	Use categories	Nur	*Nt*	Nur − *Nt*	Nur_−1_	ICF
1	Amenorrhea	57	2	55	56	0.98
2	Antiseptic	82	2	80	81	0.99
3	Breast inflammation and lactation	213	7	206	212	0.97
4	Delivery problems	84	3	81	83	0.98
5	Emmenagogue	44	1	43	43	1.00
6	Gonorrhea	199	6	193	198	0.97
7	Induce abortion	119	3	116	118	0.98
8	Labour pain and backache	100	3	97	99	0.98
9	Leucorrhoea	269	8	261	268	0.97
10	Menstrual problems	620	23	597	619	0.96
11	Prevent miscarriage	109	4	105	108	0.97
12	Sexual problems	147	5	142	146	0.97
13	Tonic after delivery	41	1	40	40	1.00
14	Vomiting stoppage	109	3	106	108	0.98

**Table 5:** Family importance value (FIV) of medicinally important families.

Sr. no.	Family name	No. of species	FC (family)	FIV
1	Acanthaceae	1	33	25.38
2	Adiantaceae	1	24	18.46
3	Alliaceae	1	25	19.23
4	Amaranthaceae	3	66	50.77
5	Anacardiaceae	1	43	33.08
6	Apiaceae	3	113	86.92
7	Asteraceae	4	100	76.92
8	Azoiaceae	1	45	34.62
9	Berberidaceae	1	45	34.62
10	Bignoniaceae	1	46	35.38
11	Brassicaceae	3	82	63.08
12	Cactaceae	1	40	30.77
13	Celastraceae	1	29	22.31
14	Chenopodiaceae	1	41	31.54
15	Convolvulaceae	1	18	13.85
16	Cucurbitaceae	1	39	30.00
17	Cyperaceae	1	33	25.38
18	Equisetaceae	1	27	20.77
19	Euphorbiaceae	2	68	52.31
20	Geraniaceae	2	74	56.92
21	Lamiaceae	7	128	98.46
22	Liliaceae	1	25	19.23
23	Malvaceae	1	40	30.77
24	Meliaceae	1	44	33.85
25	Menispermaceae	1	43	33.08
26	Mimosaceae	3	98	75.38
27	Nyctaginaceae	2	39	30.00
28	Oxalidaceae	1	37	28.46
29	Portulacaceae	1	31	23.85
30	Primulaceae	1	26	20.00
31	Rhamnaceae	2	58	44.62
32	Rosaceae	4	122	93.85
33	Sapindaceae	1	43	33.08
34	Solanaceae	3	112	86.15
35	Tamaraceae	1	42	32.31
36	Urticaceae	1	19	14.62
37	Verbenaceae	3	65	50.00
38	Zygophyllaceae	2	57	43.85

## Data Availability

The figures and tables supporting the results of this study are included within the article, and the original datasets are available from the first author or the corresponding author upon request.
